The article "Fusing Part-of-Speech Information in Low-Resource Neural Paraphrase Generation" was published in 2021. Journal: Comput Intell Neurosci.

# Fusing Part-of-Speech Information in Low-Resource Neural Paraphrase Generation

**DOI:** 10.1155/2021/9022193

**Published:** 2021-10-18

**Authors:** Xiaoqiang Chi, Yang Xiang

**Affiliations:** College of Electronics and Information Engineering, Tongji University, Shanghai 201804, China

## Abstract

Paraphrase generation is an essential yet challenging task in natural language processing. Neural-network-based approaches towards paraphrase generation have achieved remarkable success in recent years. Previous neural paraphrase generation approaches ignore linguistic knowledge, such as part-of-speech information regardless of its availability. The underlying assumption is that neural nets could learn such information implicitly when given sufficient data. However, it would be difficult for neural nets to learn such information properly when data are scarce. In this work, we endeavor to probe into the efficacy of explicit part-of-speech information for the task of paraphrase generation in low-resource scenarios. To this end, we devise three mechanisms to fuse part-of-speech information under the framework of sequence-to-sequence learning. We demonstrate the utility of part-of-speech information in low-resource paraphrase generation through extensive experiments on multiple datasets of varying sizes and genres.

## 1. Introduction

Polysemy poses a great challenge for natural language processing. In neural-network-based natural language processing models, input words are often represented as word vectors (or word embeddings). The most commonly used off-the-shelf word vectors include word2vec [1] and GloVe [2], both of which are trained on large corpora via unsupervised learning algorithms. Both embedding models present only one corresponding word vector as a dense (distributed) semantic representation for each individual word. For a word with multiple senses, its word vector is a weighted average of the representations for different senses, with the weights depending on how often the corresponding senses occur in the training corpus. An obvious drawback of this hybrid representation is that the most common sense vector representation is still used when a word is encountered in an NLP task with less common usage. It can cause significant difficulties in the learning of NLP models, including paraphrase generation.

In this work, we attempt to integrate part-of-speech information into the process of paraphrase generation. Our assumption is that different senses of a particular word could be distinguished, given the corresponding part-of-speech label or category in some cases. For instance, the word *color* in “the color of the box” and “color the wall green” would be represented by the same embedding vector by traditional methods. When given the correct part-of-speech labels (NOUN in the first phrase and VERB in the second), we could compose part-of-speech embeddings through a similar approach to word embeddings. Intuitively, when a word vector is combined with different part-of-speech embeddings, we obtain POS-specific word vectors. Hence, it could help in differentiating between various senses.

We assume POS information would help in learning better sentence representations that could, in turn, facilitate the decoding process of paraphrases, especially in low-resource conditions. To verify this hypothesis, we propose three schemes for fusing POS information in the form of POS tags into the encoder side of our paraphrase generation models. We explore two disparate network types on which encoder-decoder models are built. In particular, we consider a recurrent network that is the most widely employed architecture for sequence modeling in NLP and a self-attention-based network invented in recent years and has achieved great success in both speed and performance in various domains.

## 2. Related Work: NLP Using Part-of-Speech Information

In this section, we summarize NLP models that use part-of-speech information, a particular type of linguistic knowledge most relevant to our work.

Zhou et al. [3] used multiple lexical features of the input text as well as the location information of the answers in the task of generating relevant question sentences given a piece of text. The lexical features they used include part-of-speech labels, named entity recognition information, and word case information. These different classes of information are integrated with a concatenation approach to obtain a feature-informative hybrid word vector representation. They propose to apply a neural encoder-decoder model to generate meaningful and diverse questions from natural language sentences. The encoder reads the input texts and answer positions to produce an answer-aware input representation and feeds it to the decoder to produce an answer-centered question sentence. The model achieved a good BLEU4 score on the SQuAD [4] dataset. They also conducted ablation experiments on four different types of information and found that the model performance was most affected when the answer location information was removed, followed by named entity recognition information and part-of-speech information.

Ramesh et al. [5] applied the sequence-to-sequence (seq2seq) model to the abstractive text summarization task with an enhanced feature representation scheme for their encoder. Specifically, they used lexical features including part-of-speech labels, named entity recognition labels, TF (term frequency), and IDF (inverse document frequency). The two real-valued features, TF and IDF, were not integrated into a single feature, TF-IDF [6], but were separately involved in the representation of the word features. The TF and IDF are first discretized into a fixed number of value ranges to construct the corresponding embedding vectors and thus transformed into category values. The numbering of the ranges is their corresponding index values, which can be used to retrieve the corresponding embedding vectors in the embedding matrix. These four lexical features are concatenated onto the word vector to obtain a feature-enhanced representation of word vectors.

There are several lines of work that incorporate part-of-speech information in sentiment classification tasks. Nicholls and Song [7] performed sentiment analysis within the framework of traditional machine learning, and the model they use is the maximum entropy classifier [8, 9]. While previous models used word weights calculated from statistical information on word frequency, this paper takes part-of-speech information into account, with various part-of-speech categories having different weights. They focus on four part-of-speech categories: nouns, verbs, adjectives, and adverbs while ignoring other part-of-speech categories. The lexical strengths were taken as values from 1 to 5, resulting in 625 combinations in total. By traversing all the weight possibilities, they obtained the optimal part-of-speech strengths. Compared with the baseline model that does not consider lexical information, their proposed model has a score improvement of more than 4 percentage points in both accuracy and F1 values.

In Wang et al.'s study [10], unlike existing random subspace (RS) methods that use a single subspace rate to control the diversity of the base learners, POS-RS uses two important parameters, namely the content lexicon subspace rate and the feature lexicon subspace rate, to control the balance between accuracy and diversity of the base learners. The random subspace approach uses the subspace rate (the ratio of the number of selected features to the total number of features) to randomly select features to construct sub-datasets. In POS-RS, two parameters, that is, content lexicon subspace rate and function lexicon subspace rate, are proposed to construct sub-datasets, which can control the base learners' accuracy and diversity. The feature space is divided into content lexicon features and functional lexicon features based on part-of-speech labels. The content words considered in their paper contain four categories: nouns, verbs, adjectives, and adverbs. After constructing the sub-datasets, the base learners are trained on the different sub-datasets. The purpose of the model-building module is to learn patterns in each sub-datasets. After each base learner is trained, the final prediction scores are given through a voting mechanism to obtain the sentiment categories. Experimental results on up to ten sentiment analysis datasets show that POS-RS achieves the best performance by reducing both bias and variance compared to the base learner (e.g., support vector machine [11, 12]).

Cheng et al. [13] incorporated lexical information into the Transformer [14] model. In order to make full use of lexical information, the paper uses lexical representations in multiple network layers. A highlight of the article is that a lexical embedding matrix is first constructed based on the index of lexical labels, and then a symmetric correlation matrix is obtained by multiplying this matrix with its transpose matrix. The vector obtained by averaging the correlation matrix over the rows is multiplied with the output matrix (word vector dimension × sentence length) of a normal Transformer network with the word vector as input to obtain a lexical attention vector. Finally, this vector is concatenated with the vector obtained by averaging the lexical embedding matrix over the columns and input to a simple classifier consisting of a linear layer and Sigmoid [15] for the prediction of sentiment categories.

Zhu et al. [16] incorporated lexical information into the learning of sentence representations. They used a classical network structure like LSTM [17] to model the sequence of words in a sentence to obtain a sequence of hidden states, where each hidden state corresponds to a word in the input sentence. The final hidden state vector is then extracted, which they call structural representation. The syntactic parsing of the sentence yields a sequence of lexical labels. They make a weighted average of the hidden state sequence according to the lexical labels to obtain a vector called syntactic representation. The weight of each hidden state depends on the lexical label of the corresponding word. These weights are network parameters learned during training. Finally, the structural and syntactic representations are combined as a vector representation of the sentence. Nevertheless, the exact combination mechanism used is not given in the article. The multiple training corpora they use are sentence pairs labeled with similarity scores. For the input training set of sentence pairs, their network learns a vector representation for each sentence and then computes a similarity value for both sentence vectors. The training goal is to minimize the mean square error between the predicted and true similarity values. Typically sentence representation learning models require only unlabeled plain text, which can be easily obtained to compose a large amount of training data. Their paper requires sentence pairs with similarity scores as training data, which is an obvious limitation.

## 3. Methods

We assume linguistic information in the form of part-of-speech tags could provide a valuable signal for learning more meaningful sentence representations, and such enhanced representations, when fed into the decoding module, would produce paraphrases with higher quality. We propose multiple schemes for integrating POS information into the encoder side of our paraphrase generation models to verify this hypothesis. Specifically, we devise three POS-augmented encoders with varying strategies for fusing POS tag representations extracted from a corresponding source sentence. We explore two disparate network types on which encoder-decoder models are built. In particular, we consider a recurrent network (RNN) [18], the most widely employed architecture for sequence modeling, and a self-attention-based network (Transformer) proposed in recent years and has achieved great success in both speed and performance since its invention.

For RNN-based encoder-decoder models, we adopt bidirectional GRU (or BiGRU) [19] on the encoder side. It is common to use bidirectional networks when learning sentence representations with recurrent layers because it allows us to glean information from both directions. To ease the understanding of our newly introduced models, we first describe the syntax-agnostic encoder as a comparison baseline.

Let *X*=(*x*_1_, *x*_2_,…, *x*_*J*_) be a source sentence and *Y*=(*y*_1_, *y*_2_,…, *y*_*I*_) be its corresponding target sentence, here *J* and *I* may not be equal. Let *E*_*w*_(·) denote the embedding function for words, we have **x**_*j*_=*E*_*w*_(*x*_*j*_), ∀*j* ∈ [1, *J*]. For the *j*th position in the source sentence, hidden vectors output by the forward GRU and backward GRU are computed as [19]

(1) $$\begin{array}{c} {\overset{⟶}{h}}_{j}={\text{GRU}}_{f}\left(x_{j},{\overset{⟶}{h}}_{j-1}\right),\\ {\overset{\leftarrow }{h}}_{j}={\text{GRU}}_{b}\left(x_{j},{\overset{\leftarrow }{h}}_{j+1}\right), \end{array}$$

where GRU_*f*_ denotes the forward GRU and GRU_*b*_ denotes the backward GRU. Then the two hidden vectors are combined to form a single vector via concatenation:

(2) $$\begin{array}{c} h_{j}={\overset{⟶}{h}}_{j}\;⊕\;{\overset{\leftarrow }{h}}_{j}. \end{array}$$

The aforementioned nets from two directions can be summarized as one function [20]:

(3) $$\begin{array}{c} h_{j}={\overset{⟶}{h}}_{j}\;⊕\;{\overset{\leftarrow }{h}}_{j}={\text{GRU}}_{f}\left(x_{j},{\overset{⟶}{h}}_{j-1}\right)\;⊕\;{\text{GRU}}_{b}\left(x_{j},{\overset{\leftarrow }{h}}_{j+1}\right)\\ =\text{BiGRU}\left(x_{j},{\overset{⟶}{h}}_{j-1},{\overset{\leftarrow }{h}}_{j+1}\right). \end{array}$$

These are the formulas for the first layer. A deeper network can be composed by stacking multiple BiGRU layers:

(4) $$\begin{array}{c} h_{j}^{\left(k\right)}=\text{BiGRU}\left(h_{j}^{\left(k-1\right)},{\overset{⟶}{h}}_{j-1}^{\left(k\right)},{\overset{\leftarrow }{h}}_{j+1}^{\left(k\right)}\right), \end{array}$$

when *k*=1, **h**_*j*_^(*k* − 1)^ reduces to the embedding vector for *x*_*j*_:

(5) $$\begin{array}{c} h_{j}^{\left(k-1\right)}=h_{j}^{\left(0\right)}=x_{j}. \end{array}$$

For an encoder comprised by *K* BiRNN layers, the final output is the set of hidden vectors:

(6) $$\begin{array}{c} {\left\{h_{j}^{\left(K\right)}\right\}}_{j=1}^{J} \end{array}$$

We refer this vanilla encoder as the *base encoder*, which is shown in Figure 1.

In this section, we use the sentence in Table 1 as example:

### 3.1. Encoder

Assume the POS tag for word *x*_*j*_ is *t*_*j*_, ∀*j* ∈ [1, *J*]. Let *E*_*t*_(·) denote the embedding function for POS tags, we have **t**_*j*_=*E*_*t*_(*t*_*j*_), ∀*j* ∈ [1, *J*]. Now we describe the first layer in each of the three syntax-augmented encoders, calculations for deeper layers are similar to that of the base encoder.

#### 3.1.1. Addition Mechanism

The first and most straightforward strategy for incorporating POS information is by addition. In the addition scheme, word embeddings **x**_*j*_ and tag embeddings **t**_*j*_ are summed up:

(7) $$\begin{array}{c} x_{j}^{\text{add}}=x_{j}+t_{j}, \end{array}$$

before feeding into the first layer:

(8) $$\begin{array}{c} h_{j}^{\text{add}}=\text{BiGRU}\left(x_{j}^{\text{add}},{\overset{⟶}{h}}_{j-1}^{\text{add}},{\overset{\leftarrow }{h}}_{j+1}^{\text{add}}\right). \end{array}$$

Here “add” is short for *addition*. *j* subscripts the word position. The dimensionalities of **x**_*j*_ and **t**_*j*_ are the same (say 256), so they can be added together.  Figure 2 shows an intuitive illustration of this scheme.

#### 3.1.2. Concatenation Mechanism

In the concatenation (abbreviated as “cat” in the sequel) scheme, word embeddings and tag embeddings are concatenated:

(9) $$\begin{array}{c} x_{j}^{\text{cat}}=x_{j}\;⊕\;t_{j}, \end{array}$$

and then fed into the first layer:

(10) $$\begin{array}{c} h_{j}^{\text{cat}}=\text{BiGRU}\left(x_{j}^{\text{cat}},{\overset{⟶}{h}}_{j-1}^{\text{cat}},{\overset{\leftarrow }{h}}_{j+1}^{\text{cat}}\right). \end{array}$$

Keeping word embeddings and POS embeddings at disjunctive dimensionalities has the benefit that they will not interfere with each other. Typically, the dimensionalities of the POS embeddings are smaller than that of the word embeddings since the size of the POS tag set is tiny when compared with the word vocabulary size. An intuitive view of this encoder is illustrated in Figure 3.

#### 3.1.3. Double-Channel Mechanism

In this scheme, words and tags are consumed by separate RNN networks

(11) $$\begin{array}{c} h_{j}^{1}=\text{BiGRU}\left(x_{j},{\overset{⟶}{h}}_{j-1}^{1},{\overset{\leftarrow }{h}}_{j+1}^{1}\right), \end{array}$$

here we use the number “1” to index the word channel as channel 1. Since the size of the tag set is small, a unidirectional RNN would be adequate to model the tag sequences:

(12) $$\begin{array}{c} h_{j}^{2}=\text{GRU}\left(t_{j},h_{j-1}^{2}\right), \end{array}$$

then the above two hidden vectors are combined into one via concatenation:

(13) $$\begin{array}{c} h_{j}^{\text{dc}}=h_{j}^{1}\;⊕\;h_{j}^{2}, \end{array}$$

where “dc” stands for double channel.

A pictorial view of this mechanism is illustrated in Figure 4.

### 3.2. Decoder

For the decoder part of our model, we also employ a GRU network. Let *s*_*i*_ represent the hidden state vector at time step *i*. A context vector is calculated via an attention module, taking the set of all encoder hidden states and the previous decoder hidden state [21]:

(14) $$\begin{array}{c} c_{i}=\text{Attention}\left({\left\{{\tilde{h}}_{j}\right\}}_{j=1}^{J},s_{i-1}\right), \end{array}$$

here ${\tilde{h}}_{j}$ is chosen from the set {**h**_*j*_, **h**_*j*_^add^, **h**_*j*_^cat^, **h**_*j*_^dc^}, depending on which encoder is adopted.

The context vector and the vector for target word **y**_*i*−1_ are concatenated into one vector which is then fed into a GRU:

(15) $$\begin{array}{c} s_{i}=\text{GRU}\left(s_{i-1},c_{i}\;⊕\;y_{i-1}\right). \end{array}$$

At last, these three vectors are processed by a linear layer, and then a softmax function that follows produces a probability distribution for the next word:

(16) $$\begin{array}{c} p\left(y_{i}\right)=\text{Softmax}\left(\text{Linear}\left(s_{i}\;⊕\;c_{i}\;⊕\;y_{i-1}\right)\right). \end{array}$$

We use a greedy decoder at inference time, selecting the output token with the highest probability at each time step.

## 4. Empirical Study

### 4.1. Datasets

We investigate three paraphrase datasets; each is further split into multiple subsets with varying sizes, resulting in eight datasets in total. This procedure allows us to study the effect of data size on model performance.

#### 4.1.1. Quora

The Quora dataset (available at https://www.kaggle.com/c/quora-question-pairs), released in January 2017, is initially developed for question duplicates. Each sample in the dataset contains a question number (ID), a pair of questions, and a binary value signifying whether the pair is duplicate. If the label is “1”, the question pair is indeed paraphrases of each other. The whole set contains about 150 K samples. After randomly sampling 2 K pairs for development and 10 K for test, we sample 50 K to constitute a training set denoted as Quora50K. From Quora50K, we again sample 20 K and 10 K pairs as another two training sets, where each dataset is a randomly sampled subset of a larger dataset. The minimum frequency for building vocabulary is set to 3 for these three Quora datasets.

#### 4.1.2. ParaNMT

The ParaNMT dataset [22] is constructed by translating a large parallel corpus using NMT. Creating this large paraphrase corpus aims to learn sentence representations whose superiority is manifested in a semantic textual similarity task. However, it is also shown to be helpful in paraphrase generation tasks. A score that represents the level of similarity is associated with each paraphrase pair. The scores are evenly divided into five ranges, and sentence pairs in the highest score range show high levels of lexical overlap. Overlapping is generally not a desirable attribute because disparate sentences are deemed to be more interesting as paraphrases. So we choose the second-highest score range (0.6–0.8) for this work. We filter out noisy sentences (script available at https://github.com/chifish/preprocess) to keep the noise level in the dataset manageable. Finally, we get 2.3 million sentence pairs. We randomly sample 2 K pairs for development and 10 K for test, respectively. From the remaining sentences, we randomly sample 100 K pairs as one training set, from which we sample another 50 K to form the second ParaNMT dataset.

#### 4.1.3. COCO

MSCOCO [23] is a large-scale dataset for object detection, segmentation, and captioning, mainly adopted by the vision community. The image captioning part is produced by asking five human annotators to describe each image's most salient object or event. Although the focus and perspective of different annotators might vary, especially for cluttered images or those with a complex background, the captions generally convey the same message, making this dataset suitable for the paraphrase generation task. The standard training and validation sets contain more than 82 K and 40 K images, respectively. Following Gupta et al. [24], we discard one caption randomly from the five captions attached to each image. Thus we could obtain two paraphrase pairs from the four remaining captions. We randomly sample 2 K pairs for development and 10 K for test, respectively, from the validation set. The training set contains about 164 K pairs in total, and this full dataset is used as one training set. From the whole training set, we sample 50 K sentence pairs as another training set. From this, we again sample a smaller dataset with 20 K pairs. Hence, we have three training set for MSCOCO : COCO (full), COCO50K, and COCO20K.

### 4.2. Experiment Configuration

The experiments in this paper are conducted using PyTorch (version 1.4.0), and we also use torch text (version 0.6.0), which comes with PyTorch and provides a range of convenient text processing tools. We use spaCy (version 2.3.2) for tokenization and part-of-speech tagging, and the spaCy model we use is en-core-web-sm-2.3.1. The encoder-decoder code is based on Bastings et al.'s work [25]. We use early-stopping [26] to monitor training and mitigate overfitting on the training data. The model that obtains the highest BLEU on the validation set is saved for test. The batch size is set to 128, and sentences of similar length are put together to minimize the amount of padding and thus improve training efficiency. This bucketing process is implemented by torch text. Between layers, we apply dropouts with a probability of 0.2. To alleviate the effect of randomness, we trained each model five times, each time choosing a random seed from 42 to 46. The performance score is the average of the five runs. As the datasets considered in this chapter are relatively small, we use one layer of networks in both the encoder (bidirectional) and decoder. These settings are the same for the training of both RNN and Transformer network structures. For other settings, the configurations of the two network structures are different, and we describe them separately below:

- RNN: we use the Adam optimizer [27] with an initial learning rate of 0.001. The word embedding dimension size is set to 256, and the hidden unit size is 128. The validation set is evaluated at the end of each epoch. We used a learning rate scheduler for the optimizer: if the validation loss did not decrease in two consecutive evaluations, the learning rate was halved. The criterion for training stopping is the BLEU score, and the tolerance number is set to 5, meaning that if the BLEU score does not improve for five consecutive evaluations on the development set, training will be terminated. For the “cat” and “dc” mechanisms, the dimensionality of the tag embedding is set to 64, and the number of hidden units of the tag encoder using the “dc” mechanism is also set to 64. To keep the total dimensionality constant after combining word vector and tag vector, we set the dimensionality of the word vector of the source sentence to 256 − 64 = 192.
- Transformer: the hidden layer size is set to 256, the number of heads in the multihead self-attention mechanism is 8, and the feed-forward layer dimension size is 1024. We use the decay learning rate scheduler named Noam [14]. The number of epochs in the warmup phase is 5 (the first 5 epochs of training are the warmup phase) except the COCO dataset, which uses the first 2 epochs for warmup. For all models, the word embeddings are multiplied by a factor of $\sqrt{d}$ for scaling to prevent being overwhelmed when added with the positional embeddings, where *d* denotes the hidden layer size of the model. For the POS-enhanced model that uses an addition mechanism to integrate syntactic information, the POS label embeddings are scaled by $\sqrt[{4}]{d}$, which forces the three embedding vectors to be at different scales.

## 5. Results and Analysis

### 5.1. Prediction Scores

The three datasets were further divided into eight datasets. We evaluate the paraphrase sentences generated by various model configurations using various evaluation metrics including BLEU [28] and ROUGE [29]. The corresponding scores are shown in Tables 2to 7 . In addition, we perform significance test for the three POS-enhanced models proposed in this work against the base model: “†” indicates significantly better than base (*p* < 0.1), “††” indicates significantly better than base (*p* < 0.05) and “†††” indicates significantly better than base (*p* < 0.01).

In Table 2, all results are significant, so we omit the sign of the significance test for the sake of brevity. From the table, we can see that all three mechanisms of POS fusion show significant performance gains relative to the POS-agnostic model, especially the double-channel model (dc), which obtains a gain close to 0.5 BLEU on Quora50K. The gains are even larger when the size of the dataset decreases: the gains on Quora20K and Quora10K are about 1 BLEU and 1.4 BLEU, respectively. A similar pattern can be observed for the other evaluation metrics.

In Table 3, most of the results are significant. When the data size is large, fusing lexical information in another channel does not necessarily improve the model's performance. There is a slight decrease in the corresponding BLEU values in the table. However, we can see at the same time that the other evaluation metrics still show a significant improvement. The improvement obtained by the three POS fusion mechanisms is significant in all metrics when the data size is reduced to half. It can also be seen from the table that for the ParaNMT datasets, the simpler addition mechanism (add) and the concatenation mechanism (cat) perform better than the double-channel mechanism (dc).

As can be seen in Table 4, when the data size is large (COCO sample size is about 165 K), fusing lexical information has almost no effect on the model performance. As the size of the dataset decreases, the value of lexical information begins to emerge. At a training set size of 20 K, the double-channel mechanism achieves significant improvements in all metrics.

In Table 5, significance levels for all scores are *p* < 0.01, except for the ROUGE-1 and ROUGE-L scores on the Quora20K dataset, where the significance level for the double-channel mechanism is *p* < 0.05. The fact that the lexical enhancement model still achieves a significant boost on Transformer, a stronger baseline than RNN, adds further evidence to the effectiveness of the lexical fusion mechanism. Looking at the results of each dataset in the table together, we find that the concatenation mechanism shows the best performance.

In Table 6, we can see that the concatenation mechanism shows significantly better performance than the base model in all metrics except BLEU. For the addition mechanism, on the contrary, the advantage becomes obvious on smaller datasets. A noteworthy point is that the performance of the baseline model exhibits huge fluctuations at a dataset size of 50 K, as can be seen from the standard deviations in parentheses that follow. For example, the standard deviation of the corresponding BLEU value is 0.47. This fluctuation causes some difficulty in comparing significance levels, making it impossible to reach significance levels even when the mean BLEU values of the addition and concatenation mechanisms are 0.3 higher than those of the baseline model. The advantage of the double-channel mechanism is not as apparent as simpler mechanisms, and this pattern can also be observed in Table 7.

### 5.2. Effect of Sentence Length

Including sentences with a length beyond 15 allows us to study another dimension of syntax-enhanced models: the effect of sentence length on model performance. To this end, we split the sentences predicted by models trained on each Quora dataset into six buckets according to the lengths of source sentences and compute BLEU scores for each separate bucket. We choose the Quora datasets for analysis because Quora is the most widely investigated paraphrase dataset and omits other datasets' analyses for space considerations.

Results for RNN-based models are illustrated in Figure 5. Results for Transformer-based models are illustrated in Figure 6.

### 5.3. Analysis

As can be seen in Figure 5(a), the lexically enhanced models show significantly better performance than the baseline for sentences with length up to 20. The double-channel mechanism shows the most significant advantage: a clear margin in all length ranges. The spike for the 21 to 25 length range is notable and quite unexpected: all models show unusually high scores, including the baseline model. We hypothesize that this is due to the nature of the dataset itself: the data distributions on source and target sides for this range are most similar, resulting in an easy subset for paraphrase models. To verify this, we divided the Quora50K training and test sets by length and calculated several distribution statistics. The results are shown in Figure 7.

Figure 7(a) shows the BLEU values calculated from the dataset itself, which is equivalent to using the source sentence as the predicted sentence to calculate the BLEU, and the reference sentence remains the real target sentence. The score reflects the surface similarity to some extent, that is, the degree of overlap, between the source and target sentences. Higher scores indicate that the source and target sentences in this length interval are more similar to each other, and the corresponding sentence pairs are simpler for the paraphrase generation model and thus easier to generate. The score for the 21 to 25 length interval is unusually high, which explains the corresponding curve in the previous illustration.

To have a clearer understanding of the characteristics of the dataset, we further analyzed the metrics related to its length distribution.  Figure 7(b) depicts the distribution of the length ratio between the source and target sentences, which is calculated by taking the larger of the two lengths as the numerator and then take the average in each interval so that the value is greater or equal to 1. This ratio reflects the degree of alignment of the corpus to a certain extent. Generally speaking, the closer the ratio is to 1, the better the alignment of the corpus is. This length ratio reflecting the degree of alignment is usually used in bilingual parallel corpus filtering strategies, and it is generally believed that sentence pairs with too high a ratio (e.g., greater than 1.5) contain too much noise and are not beneficial to the training of translation models.

From Figure 7(b), we can easily observe that the length ratio of intervals located at both ends is relatively high, which reflects the low alignment of sentence pairs in the corresponding intervals, bringing some difficulties for the model to learn. In particular, the average length ratio on the test set for the shortest interval (≤5) even exceeds 1.7 and is nearly 0.2 higher than the ratio on the training set. This mismatch between the ratios on the training and test sets also poses a challenge for model inference.

Another metric related to the length distribution is the length distribution of the source sentences, as shown in Figure 7(c). We also give the corresponding distribution on the test set, which helps understand how the model performs on the test set.

The sentence length distribution illustrated in Figure 7(c) shows that the length distribution in the Quora dataset is highly unbalanced. Most of the sentences are concentrated in the 6 to 10 and 11 to 15 length intervals. In particular, the 6 to 10 interval accounts for more than 50% of the sentences in both the training and test sets. In contrast, the intervals located at the two ends of the spectrum take up only a tiny fraction, and the 26 to 30 interval represents a share of less than 1%. This sparsity of data poses another challenge to the learning of the model. In addition, we note that there is a significant difference in the length distribution between the training and test sets on the shortest interval (≤5): the test set has about three times the proportion of the training set in this interval. This mismatch between the training and test sets also poses a challenge for model inference. Combining the ratio distribution in Figure 7(b) and the length distribution in Figure 7(c), we can infer that the length intervals located at the two ends (≤5 and 26–30) belong to the more difficult data subsets, which could explain the low BLEU scores of each model at both ends of the curves in Figures 5 and 6.

## 6. Conclusion

Syntactic information is typically ignored in the process of neural paraphrase generation. The underlying assumption is that neural networks could learn such information (and other features) implicitly. We explored the possibility of augmenting sequence-to-sequence paraphrase generation models with explicit syntax information in the form of part-of-speech tags. This augmentation is an extension to feature representation in sequence to sequence learning, which has been shown to be effective for a wide spectrum of natural language generation tasks. Specifically, we explore two common network architectures, RNN, and Transformer, and investigate three strategies for combining part-of-speech embedding with word embedding, respectively.

Experiments on various datasets show the effectiveness of part-of-speech information, and the advantages of our proposed models are more significant under low-resource conditions. Taking the Quora50K dataset as an example, the boosts of BLUE scores in the RNN-based model relative to the baseline model for the addition, concatenation, and double-channel mechanisms are 1.56%, 1.31%, and 2.14%, respectively; in the Transformer-based model, the corresponding boosts are 2.22%, 2.67%, and 1.69%, respectively. As for the Quora10K dataset, the improvement of BLUE values in the RNN-based model relative to the baseline model reached 5.59%, 4.35%, and 9.16% for the addition, concatenation, and double-channel mechanisms, respectively; and the corresponding improvement reached 3.08%, 4.03%, and 4.33% in the Transformer-based model, respectively.

The approach for augmenting paraphrase generation models with syntactic information proposed herein is convenient and straightforward to implement. Hence, it could be easily adapted to other paraphrase generation models (and other language generation models in general) that do not take into account linguistic knowledge (syntax information in particular). We hope our work could inspire other researchers to exploit similar information. No POS taggers provide perfect predictions, thus using POS information would introduce inaccuracies into NLP models. Tackling this issue (by adopting fuzzy logic-based techniques [30,31], for instance) could be considered a direction for future research. Leveraging both POS labels and syntax information such as dependency parses [32] in paraphrase generation models is also a potential direction for further study.

## Figures and Tables

**Figure 1:** The “base” encoder.

**Figure 2:** The “add” encoder.

**Figure 3:** The “cat” encoder.

**Figure 4:** The “dc” encoder.

**Figure 5:** Performance comparison between RNN-based models per source sentence length for Quora datasets: (a) results on Quora10K, (b) results on Quora20K, and (c) results on Quora50K.

**Figure 6:** Performance comparison between Transformer-based models per source sentence length for Quora datasets: (a) results on Quora10K, (b) results on Quora20K, and (c) results on Quora50K.

**Figure 7:** Dataset statistics for Quora datasets: (a) BLEU score computed between source and target sentences on Quora50K and Quora test set, (b) average ratio between the lengths of the longer sentence and the shorter sentence in source-target pairs, and (c) proportion each range represents.

**Table 1:** Example of part-of-speech tag.

word	How	to	stop	smoking	?
tag	WRB	TO	VB	VBG	.

**Table 2:** Performance of RNN-based models on Quora datasets.

Dataset	Model	BLEU	ROUGE-1	ROUGE-2	ROUGE-L
Quora10K	base	15.39 (±0.22)	38.47 (±0.29)	20.54 (±0.24)	37.43 (±0.26)
	add	16.25 (±0.08)	39.82 (±0.23)	21.53 (±0.15)	38.77 (±0.22)
	cat	16.06 (±0.04)	39.51 (±0.09)	21.27 (±0.09)	38.46 (±0.09)
	dc	16.8 (±0.13)	40.79 (±0.3)	22.02 (±0.24)	39.64 (±0.32)

Quora20K	base	17.8 (±0.16)	43.52 (±0.21)	24.08 (±0.17)	42.12 (±0.19)
	add	18.34 (±0.09)	44.42 (±0.13)	24.73 (±0.12)	43.01 (±0.12)
	cat	18.21 (±0.12)	44.12 (±0.06)	24.52 (±0.04)	42.73 (±0.06)
	dc	18.79 (±0.25)	45.26 (±0.22)	25.31 (±0.31)	43.82 (±0.21)

Quora50K	base	20.57 (±0.12)	48.63 (±0.15)	28.12 (±0.15)	46.84 (±0.13)
	add	20.89 (±0.11)	49.1 (±0.06)	28.4 (±0.1)	47.27 (±0.08)
	cat	20.84 (±0.05)	48.95 (±0.08)	28.36 (±0.1)	47.13 (±0.07)
	dc	21.01 (±0.1)	49.61 (±0.12)	28.82 (±0.13)	47.81 (±0.08)

**Table 3:** Performance of RNN-based models on ParaNMT datasets.

Dataset	Model	BLEU	ROUGE-1	ROUGE-2	ROUGE-L
ParaNMT50K	base	10.96 (±0.07)	35.12 (±0.13)	14.7 (±0.1)	32.84 (±0.14)
	add	11.27 (±0.1)^†††^	35.75 (±0.16)^†††^	15.1 (±0.11)^†††^	33.44 (±0.14)^†††^
	cat	11.24 (±0.07)^†††^	35.54 (±0.12)^†††^	15.0 (±0.11)^†††^	33.28 (±0.13)^†††^
	dc	11.09 (±0.16)^†^	35.85 (±0.51)^††^	15.05 (±0.37)^†^	33.56 (±0.5)^††^

ParaNMT100K	base	12.35 (±0.13)	38.98 (±0.12)	16.99 (±0.12)	36.29 (±0.1)
	add	12.6 (±0.12)^†††^	39.4 (±0.24)^†††^	17.36 (±0.16)^†††^	36.72 (±0.23)^†††^
	cat	12.59 (±0.08)^†††^	39.31 (±0.11)^†††^	17.26 (±0.09)^†††^	36.62 (±0.1)^†††^
	dc	12.3 (±0.13)	39.35 (±0.11)^†††^	17.17 (±0.1)^††^	36.64 (±0.1)^†††^

**Table 4:** Performance of RNN-based models on COCO datasets.

Dataset	Model	BLEU	ROUGE-1	ROUGE-2	ROUGE-L
COCO20K	base	6.15 (±0.23)	35.32 (±0.22)	10.86 (±0.23)	29.71 (±0.18)
	add	6.2 (±0.14)	35.77 (±0.11)^†††^	11.01 (±0.06)	30.03 (±0.07)^†††^
	cat	6.27 (±0.21)	35.74 (±0.15)^†††^	11.04 (±0.18)	30.01 (±0.17)^††^
	dc	6.4 (±0.05)^††^	35.8 (±0.26)^††^	11.46 (±0.15)^†††^	30.36 (±0.27)^†††^

COCO50K	base	6.9 (±0.04)	37.41 (±0.2)	12.02 (±0.16)	31.42 (±0.12)
	add	6.99 (±0.2)	37.54 (±0.14)	12.19 (±0.07)^††^	31.6 (±0.09)^††^
	cat	6.92 (±0.19)	37.6 (±0.09)^†^	12.11 (±0.12)	31.58 (±0.08)^††^
	dc	6.99 (±0.1)^†^	37.56 (±0.21)	12.44 (±0.18)^†††^	31.76 (±0.19)^†††^

COCO	base	7.68 (±0.03)	39.18 (±0.17)	13.11 (±0.1)	32.95 (±0.09)
	add	7.61 (±0.14)	39.15 (±0.18)	13.13 (±0.11)	32.91 (±0.12)
	cat	7.55 (±0.15)	39.13 (±0.15)	13.02 (±0.13)	32.89 (±0.14)
	dc	7.62 (±0.09)	39.21 (±0.15)	13.3 (±0.13)^††^	33.03 (±0.05)^†^

**Table 5:** Performance of Transformer-based models on Quora datasets.

Dataset	Model	BLEU	ROUGE-1	ROUGE-2	ROUGE-L
Quora10K	base	20.11 (±0.11)	48.84 (±0.17)	27.28 (±0.17)	47.57 (±0.18)
	add	20.73 (±0.15)	49.82 (±0.16)	28.17 (±0.16)	48.56 (±0.16)
	cat	20.92 (±0.11)	50.47 (±0.26)	28.72 (±0.22)	49.17 (±0.25)
	dc	20.98 (±0.09)	49.49 (±0.15)	28.12 (±0.16)	48.26 (±0.15)

Quora20K	base	22.07 (±0.12)	52.09 (±0.21)	29.91 (±0.2)	50.53 (±0.18)
	add	22.41 (±0.12)	52.82 (±0.13)	30.46 (±0.11)	51.21 (±0.14)
	cat	22.71 (±0.23)	53.24 (±0.21)	30.87 (±0.23)	51.65 (±0.2)
	dc	22.64 (±0.18)	52.43 (±0.2)^††^	30.39 (±0.2)	50.92 (±0.21)^††^

Quora50K	base	24.3 (±0.1)	56.02 (±0.08)	33.07 (±0.09)	54.1 (±0.07)
	add	24.84 (±0.14)	56.58 (±0.18)	33.59 (±0.16)	54.66 (±0.18)
	cat	24.95 (±0.26)	56.8 (±0.07)	33.86 (±0.1)	54.88 (±0.04)
	dc	24.71 (±0.15)	56.25 (±0.11)	33.44 (±0.08)	54.41 (±0.09)

**Table 6:** Performance of Transformer-based models on ParaNMT datasets.

Dataset	Model	BLEU	ROUGE-1	ROUGE-2	ROUGE-L
ParaNMT50K	base	13.7 (±0.47)	41.7 (±0.66)	19.29 (±0.5)	39.54 (±0.65)
	add	14.04 (±0.2)	42.37 (±0.15)^††^	19.68 (±0.21)	40.18 (±0.17)^††^
	cat	14.05 (±0.17)	42.55 (±0.23)^††^	19.77 (±0.17)	40.34 (±0.24)^††^
	dc	13.84 (±0.07)	41.97 (±0.09)	19.4 (±0.06)	39.78 (±0.08)

ParaNMT100K	base	15.8 (±0.23)	45.5 (±0.21)	22.01 (±0.21)	43.03 (±0.22)
	add	15.85 (±0.19)	45.76 (±0.3)^†^	22.14 (±0.25)	43.3 (±0.27)^†^
	cat	15.94 (±0.06)	46.09 (±0.17)^†††^	22.34 (±0.09)^†††^	43.58 (±0.12)^†††^
	dc	15.38 (±0.1)	45.28 (±0.06)	21.69 (±0.09)	42.76 (±0.08)

**Table 7:** Performance of Transformer-based models on COCO datasets.

Dataset	Model	BLEU	ROUGE-1	ROUGE-2	ROUGE-L
COCO20K	base	7.85 (±0.1)	38.18 (±0.09)	13.94 (±0.07)	35.33 (±0.05)
	add	8.05 (±0.11)^††^	38.4 (±0.18)^††^	14.16 (±0.13)^†††^	35.49 (±0.15)^††^
	cat	8.16 (±0.1)^†††^	38.65 (±0.17)^†††^	14.29 (±0.06)^†††^	35.57 (±0.2)^††^
	dc	7.88 (±0.11)	38.27 (±0.08)^†^	13.96 (±0.11)	35.28 (±0.11)

COCO50K	base	8.34 (±0.09)	39.79 (±0.08)	14.84 (±0.05)	36.48 (±0.04)
	add	8.5 (±0.16)^†^	40.04 (±0.17)^††^	15.07 (±0.12)^†††^	36.68 (±0.11)^†††^
	cat	8.56 (±0.08)^†††^	40.0 (±0.06)^†††^	15.08 (±0.06)^†††^	36.58 (±0.06)^††^
	dc	8.21 (±0.2)	39.69 (±0.21)	14.77 (±0.17)	36.43 (±0.11)

COCO	base	8.92 (±0.16)	41.15 (±0.28)	15.74 (±0.2)	37.63 (±0.19)
	add	9.1 (±0.09)^††^	41.51 (±0.09)^††^	15.98 (±0.1)^†††^	37.83 (±0.08)^††^
	cat	9.12 (±0.19)^†^	41.46 (±0.24)^†^	15.97 (±0.19)^†^	37.8 (±0.17)
	dc	8.84 (±0.19)	41.13 (±0.26)	15.67 (±0.2)	37.58 (±0.2)

## Data Availability

The datasets investigated in this work are publicly available at https://www.kaggle.com/c/quora-question-pairs, https://drive.Google.com/file/d/1rbF3daJjCsa1-fu2GANeJd2FBXos1ugD/view, and https://cocodataset.org/#home.
